The article "Comprehensive Analysis of the Immune Implication of AKAP12 in Stomach Adenocarcinoma" was published in 2022. Journal: Comput Math Methods Med.

# Comprehensive Analysis of the Immune Implication of AKAP12 in Stomach Adenocarcinoma

**DOI:** 10.1155/2022/3445230

**Published:** 2022-09-13

**Authors:** Zhiquan Xu, Ling Xiang, Linglong Peng, Haitao Gu, Yaxu Wang

**Affiliations:** ^1^Department of Gastrointestinal Surgery, The Second Affiliated Hospital of Chongqing Medical University, Chongqing 400010, China; ^2^Department of Clinical Nutrition, The Second Affiliated Hospital of Chongqing Medical University, Chongqing 400010, China

## Abstract

A kinase anchor protein 12 (AKAP12) as a tumor suppressor in various cancers has been extensively studied and confirmed. However, its immune implication in stomach adenocarcinoma (STAD) remains uncertain. Here, using The Cancer Genome Atlas (TCGA), Human Protein Atlas (HPA), Tumor Immune Estimation Resource (TIMER), Cancer Cell Line Encyclopedia (CCLE), integrated repository portal for tumor-immune system interactions (TISIDB), and Search Tool for the Retrieval of Interaction Gene/Proteins (STRING) database, we systematically analyzed the immune correlation of AKAP12 from three aspects including immune infiltration cells, immune-related pathways, and immunomodulators and developed a AKAP12-related 4-gene signature for prognosis prediction. Our results showed that AKAP12 mRNA and protein levels were downregulated in STAD patients, and its expression was positively related to CD4+ T cells and macrophages. In addition, the immune cell infiltration levels were associated with AKAP12 gene copy number deletion in STAD. Based on CCLE database, we found that AKAP12 coexpressed genes were enriched in several immune- and cancer-related pathways, which was further validated by Gene Set Enrichment Analysis (GSEA). Moreover, we identified 46 immunomodulators that were significantly related to AKAP12 expression using TISIDB database, and these immunomodulators were involved in immune-related pathways including Th17 cell differentiation and natural killer cell-mediated cytotoxicity. Additionally, based on the 46 AKAP12-related immunomodulators, a 4-gene risk prediction signature was developed using the Cox regression model. The risk signature was identified as an independent prognostic factor, which can accurately predict the prognosis of patients with STAD, showing good predictive performance. Furthermore, we constructed a prognostic nomogram and calibration to predict and assess patient survival probabilities by integrating the risk score and other clinical factors. In conclusion, our study provides strong evidence that AKAP12 is closely related to tumor immunity in STAD from three aspects: immune infiltration cells, immune pathways, and immunomodulators. More importantly, the AKAP12-related prognostic signature may have a good application prospect for clinical practice.

The article "Comprehensive Analysis of the Immune Implication of AKAP12 in Stomach Adenocarcinoma" was published in 2022. Journal: Comput Math Methods Med.

## 1. Introduction

Stomach adenocarcinoma (STAD) is the fifth most common malignant tumor and one of the main causes of cancer deaths, accounting for 7.7% of all cancer deaths [1]. Its occurrence is a progressive process involving multiple steps and multiple factors, such as environmental diet, helicobacter pylori infection, heredity, and precancerous state. In the early stage of STAD, there are only some unclear upper gastrointestinal symptoms, such as abdominal pain, anorexia, and mild anemia. With the progress of the disease, pyloric or cardiac obstruction may occur, and complications such as upper gastrointestinal hemorrhage and perforation may also occur. Local masses, ascites, and supraclavicular lymph node enlargement can be seen in advanced STAD. At present, surgery is the main treatment for gastric adenocarcinoma. Chemotherapy, radiotherapy, and traditional Chinese medicine can be used as auxiliary treatments. Clinically, for resectable STAD patients, the comprehensive treatment model based on surgical resection combined with chemotherapy has certain curative effects, but the tumor is prone to progress or relapse, and the 5-year survival rate of advanced STAD patients is as low as 10% to 15% [2]. For unresectable and metastatic STAD, patients can obtain limited benefit from typical therapies, including systemic chemotherapy and targeted drugs, but they are facing a larger treatment bottleneck, and the survival time of patients usually does not exceed 1 year [3]. Although the individualized comprehensive treatment strategy based on surgery has been widely used in STAD, tumor recurrence and metastasis are still the main reasons for its high mortality. Moreover, the early diagnosis rate of STAD is low. Most patients with STAD have been in local progression stage when they visit the hospital, and the direct surgical effect is not ideal. Therefore, novel treatment strategies and biomarkers are urgently needed.

Recently, the emergence of immune checkpoint inhibitors (ICI) has officially kicked off the era of tumor immunotherapy. As a new type of treatment, tumor immunotherapy is based on the human immune system to exert antitumor effects by inhibiting negative feedback immune regulation mechanisms [4]. Immune checkpoint regulation is one of the most important immune regulation mechanisms for antitumor treatment, which regulates the intensity or breadth of the immune response through ligand-receptor binding [5]. Programmed cell death 1(PD-1) and programmed cell death ligand 1 (PD-L1) are the most well-known target molecules for immune checkpoint blockade [6]. PD-1/PD-L1 pathway inhibitors have achieved significant clinical effects in the treatment of a variety of malignant tumors such as melanoma, bladder cancer, lung cancer, and renal cell carcinoma [7]. Especially, PD-L1 expression is upregulated in gastric cancer and is closely related to tumor progression and patient prognosis [8]. Moreover, in several clinical trials, ICI alone or in combination with other treatment options have achieved good positive results and less toxic side effects for STAD [9–11]. Thus, some ICI were used in clinical. For instance, trastuzumab is used for human EGFR-2 positive gastric cancer, and pembrolizumab is used for second-line and later-line treatment of gastric cancer with highly microsatellite instability/different mismatch repair (MSI-H/dMMR) [10, 11]. However, the effective response rate for immunotherapy is limited to fraction of gastric cancer patients, and the commonly used markers, such as PD-L1, tumor mutation burden and tumor infiltrating leukocytes, also have certain defects in assessing the response to immunotherapy [12]. Therefore, it is essential to identify novel biomarker and to explore its immune implication, thus enhancing individualized treatment and improving the success rate of immunotherapy. In silico analysis is promising to screen out useful biomarkers for immune therapy. For example, Wang and his colleagues screened immune-associated DEGs between esophageal cancer and normal samples using TCGA and immPORT databases, based on which a 6-immune gene prognostic model was constructed by regression algorithm and examined both in survival and immunity terms [13]. Similarly, the current study was processed bioinformatically on the role of AKAP12 in the immunity of stomach carcinoma.

The article "Comprehensive Analysis of the Immune Implication of AKAP12 in Stomach Adenocarcinoma" was published in 2022. Journal: Comput Math Methods Med.

A kinase anchor protein 12 (AKAP12), as an intracellular macromolecular scaffold protein and a member of kinase anchoring proteins family, participates in the integrated regulation of multiple signals in biological cells and exert an important role in maintaining the integrity of normal tissue structure and function by anchoring protein kinase C, protein kinase A, F-actin, etc. [14]. In recent years, a series of studies have reported that AKAP12 expression is downregulated in many types of tumors, such as liver cancer, colorectal cancer, prostate cancer, and lung cancer [15]. Its decreased expression and low activity in tumor cells may be due to hypermethylation in the promoter region of AKAP12 gene and are closely related to the malignancy degree [16, 17]. Moreover, the vitro and vivo experiments have confirmed that overexpression of AKAP12 significantly inhibits tumor cell proliferation and metastasis by controlling oncogenic signaling pathways in a spatiotemporal manner [18]. In contrast, tumor malignant biological behaviors were enhanced by interfering with the expression of AKAP12 [19, 20]. The occurrence of tumor is determined by the interaction between tumor cells and the tumor microenvironment including immune infiltrating cell microenvironment around tumor cells [21]. However, as a well-known tumor suppressor, the immune implication of AKAP12 in STAD has not been explored.

The article "Comprehensive Analysis of the Immune Implication of AKAP12 in Stomach Adenocarcinoma" was published in 2022. Journal: Comput Math Methods Med.

In the present study, comprehensive bioinformatics analysis was performed to evaluate the association between AKAP12 expression and immune infiltration cells, immunomodulators, and the signaling pathways regulating the AKAP12-mediated immune response. Moreover, based on AKAP12-associated immunomodulators, we developed a 4-immunomodulator prognostic signature for survival prediction in STAD. In this step, we used univariate and multivariate Cox regression analyses to construct and validate prognostic characteristics and evaluate the predictive performance of risk scores, etc. Cox regression analysis takes survival outcome and survival time as dependent variables and can simultaneously analyze the impact of many factors on survival. Because of its excellent nature, it has been widely used in medical follow-up studies.

## 2. Materials and Methods

### 2.1. Data Collection

The transcriptome profiling (type: HTSeq–FPKM) and clinical information (type: bcr xml) of STAD were both downloaded from The Cancer Genome Atlas (TCGA) project (https://portal.gdc.cancer.gov/). A total of 407 RNA expression profile samples were obtained, which included 375 tumor samples and 32 normal samples. The clinical data of 443 STAD cases were downloaded. After excluding patients with missing survival data and crucial clinical factors, the information of 371 samples was retained for further analysis.

### 2.2. AKAP12 Expression Analysis

Difference analysis of AKAP12 mRNA expression in normal and STAD samples was performed by R package “limma.” The immunohistochemical protein expression of AKAP12 gene in normal and STAD samples was obtained from the Human Protein Atlas (HPA) database (https://www.proteinatlas.org/) [22].

### 2.3. Correlation Analysis between AKAP12 and Immune Cell Based on Tumor Immune Estimation Resource (TIMER) and CIBERSORT

TIMER database contains three modules: immune association, cancer exploration, and immune estimation, and it is a reliable tool to investigate the relationship between immune infiltration and target gene (https://cistrome.shinyapps.io/timer/) [23]. In this study, the correlations between AKAP12 expression levels/copy number alterations (CNA) and six types of immune cells were estimated using the TIMER “immune association” modules. CIBERSORT is an R/web version tool that deconvolves the expression matrix of human immune cell subtypes based on the principle of linear support vector regression [24]. This method is based on a known reference gene set and provides a set of gene expression characteristics of 22 immune cell subtypes, namely, LM22 [25]. In our study, we used CIBERSORT to calculate the abundance of immune cells in TCGA-STAD samples based on LM22, and samples were assigned into AKAP12^high^ and AKAP12^low^ groups according to AKAP12 expression medium. Difference analysis of 22 types of immune cells between the two groups was performed by R package “limma” and visualized by R package “vioplot.”

The article "Comprehensive Analysis of the Immune Implication of AKAP12 in Stomach Adenocarcinoma" was published in 2022. Journal: Comput Math Methods Med.

### 2.4. Analysis and Validation of Immune-Related Pathways of AKAP12 Coexpressed Genes

To investigate AKAP12-related pathways, we first downloaded the RNA-seq data of 37 stomach cancer cell lines from the Cancer Cell Line Encyclopedia (CCLE) website (https://sites.broadinstitute.org/ccle) and processed them by perl [26]. Based on the expression matrix data of stomach cell lines, we further screened out AKAP12 coexpressed genes through the “limma” R package with the filtering conditions: correlation coefficient > 0.5 and *p* value < 0.05. Finally, these coexpressed genes were subjected to Kyoto Encyclopedia of Genes and Genomes (KEGG) and Gene Ontology (GO) enrichment analyses with the filtering condition *p* value < 0.05, which was visualized by the “ggplot2” R package. To further clarify the gene set related to AKAP12, the medium expression value of AKAP12 divided 37 stomach cancer cell lines into AKAP12^high^ and AKAP12^low^ groups, and Gene Set Enrichment Analysis (GSEA) was performed by setting the predefined gene sets “c2.cp.kegg.v7.4.symbols.gmt” with false discovery rate (FDR) *p* value < 0.05 and permutation value 1000 [27].

### 2.5. Analysis of AKAP12-Associated Immunomodulators

Integrated repository portal for tumor-immune system interactions (TISIDB) is a powerful website containing a large amount of tumor immunity related data, in which the association between genes and immune functions (such as lymphocytes, immunomodulators, and chemokines) for 30 types of TCGA cancers was precalculated (http://cis.hku.hk/TISIDB/) [28]. In this study, we used TISIDB to identify AKAP12 expression-associated immunostimulators and immunoinhibitors under the condition *p* value < 0.05 through Spearman correlation test. Then, AKAP12-associated immunomodulators were used to construct a protein-protein interaction (PPI) network using Search Tool for the Retrieval of Interaction Gene/Proteins (STRING) database (https://string-db.org/) with setting high confidence at 0.7 [29]. Afterward, AKAP12-associated immunomodulators were subjected to GO and KEGG analysis using WebGestalt online tool (http://www.webgestalt.org/) with FDR < 0.05 [30].

The article "Comprehensive Analysis of the Immune Implication of AKAP12 in Stomach Adenocarcinoma" was published in 2022. Journal: Comput Math Methods Med.

### 2.6. Construction of the Prognostic Signature and Nomogram

The association of AKAP12-associated immunomodulators and prognosis was analyzed by stepwise Cox regression analysis using R package “survmine” and “glmnet.” A prognostic signature was established based on the AKAP12-associated immunomodulators. According to the multivariate Cox result, the risk score for each patient was calculated through the formula: risk score = *β*1*x*1 + *β*2*x*2 + ⋯+*βixi*, where *βi* represents the coefficient of each prognostic gene, and *xi* represents the expression level of prognostic gene [31]. The association between risk score and survival time was determined by Kaplan–Meier survival curve and log-rank test. Multivariate Cox regression analysis was used to assess the independence of risk score from other clinical factors. The prediction performance of risk score was evaluated using R package “survivalROC.” The nomogram was constructed to predict the impact of important clinical parameters including risk score on the overall survival of patients using R package “rms,” and the consistency index (C-index) is calculated to evaluate the prediction accuracy of the nomogram [32]. Calibration curves were plotted to compare the predicted survival rate with actual survival rate by R package “rms.”

### 2.7. Statistical Analysis

Statistical analyses were conducted by R (v4.0.5). Student's *t*-test was used to compare differences between groups. Survival curves were generated using the Kaplan–Meier method. Correction analysis of gene expression was performed by Spearman method. Univariate and multivariate analyses were conducted using Cox regression models to determine the independent prognostic factors. *p* value < 0.05 indicated statistical significance.

## 3. Results

### 3.1. Association between AKAP12 and Immune Infiltration Cells in STAD

As a tumor suppressor, AKAP12 mRNA and protein levels were downregulated in STAD patients (Figures 1(a) and 1(b)). We next investigate whether AKAP12 expression and copy number alterations were associated with tumor immune infiltration based on TIMER database. As shown in Figure 1(c), AKAP12 expression was positively related with infiltration levels of CD4+ T cell (cor = 0.408) and macrophage (cor = 0.545). Besides that, with chromosome arm-level deletion of AKAP12, infiltration levels of B cells, CD8+ T cells, CD4+ T cells, and dendritic cells were significantly decreased (Figure 1(d)). To further clarify the relationship between AKAP12 expression and specific immune infiltration cells, CIBERSORT method was used to determine the infiltrating fraction of 22 types of immune cells in TCGA-STAD samples, and all samples were divided into AKAP12^high^ and AKAP12^low^ expression groups based on AKAP12 expression median. Our results showed that the infiltrating proportions of plasma cells, memory activated CD4 T cells, follicular helper T cells, resting NK cells, and neutrophils were significantly higher in the AKAP12^low^ expression group (Figure 1(e)). On the contrary, patients with high AKAP12 expression displayed higher infiltrating proportions of native B cells, memory resting CD4 T cells, regulatory T cells, activated NK cells, monocytes, and resting mast cells (Figure 1(e)). The above results indicate that the expression of AKAP12 and the alteration of copy number may affect the infiltration level of tumor immune cells.

The article "Comprehensive Analysis of the Immune Implication of AKAP12 in Stomach Adenocarcinoma" was published in 2022. Journal: Comput Math Methods Med.

### 3.2. AKAP12 Is Associated with Immune-Related Pathways in Gastric Cancer

To investigate the functional and pathway enrichment of the AKAP12-associated genes, we performed the GO and KEGG analyses of the AKAP12 coexpressed genes. We first analyzed the RNA-seq data containing 37 stomach cancer cell lines from the CCLE datasets. Based on the expression matrix data of stomach cell lines, we further filtered out a series of AKAP12 coexpressed genes by setting the filtering conditions: correlation coefficient > 0.5 and *p* value < 0.05. GO results of these coexpressed genes are shown in Figure 2(a), and KEGG analysis showed that AKAP12-related coexpressed genes were enriched in cancer- and immune-related pathways, including EGFR tyrosine kinase inhibitor resistance, Ras signaling pathway, FoxO signaling pathway, p53 signaling pathway, Fc gamma R-mediated phagocytosis, PI3K-Akt signaling pathway, and mTOR signaling pathway (Figure 2(b)). Furthermore, based on the expression medium value of AKAP12 in CCLE datasets, stomach cell lines were assigned into AKAP12^high^ and AKAP12^low^ groups. As shown in Figure 2(c), GSEA enrichment analysis demonstrated that several cancer- and immune-related pathways, such as hedgehog signaling pathway, pathway in cancer, and antigen processing and presentation, were activated in the AKAP12^high^ group, which further validated that AKAP12 may affect tumor progression through immune-related pathways in gastric cancer.

### 3.3. AKAP12 Is Associated with Immunomodulators in Gastric Cancer

We next aimed to explore the relationship between AKAP12 and immunomodulators. For this purpose, TISIDB, an integrated repository portal for tumor-immune system interactions, was used to analyze the relations between immunomodulators and AKAP12 expression. Here, 15 immunoinhibitors (ADORA2A, BTLA, CD96, CD160, CSF1R, HAVCR2, IL10, IL10RB, KDR, LGALS9, PDCD1LG2, PVRL2, TGFB1, TGFBR1, and TIGIT) (Figure 3(a)) and 31 immunostimulators (C10orf54, CD27, CD28, CD40LG, CD48, CD86, CD276, CXCL12, CXCR4, ENTPD1, HHLA2, IL2RA, IL6, IL6R, KLRC1, KLRK1, MICB, NT5E, PVR, RAET1E, TMEM173, TNFRSF9, TNFRSF13B, TNFRSF13C, TNFRSF14, TNFRSF25, TNFSF4, TNFSF13, TNFSF13B, TNFSF14, and TNFSF18) (Figure 3(b)) were identified as either positively or negatively correlated with AKPA12 expression. By constructing a PPI network of the 46 immunomodulators, we obtain a close interaction relationship between AKAP12-related immunoregulatory genes (Figure 4(a)). GO function annotations showed that AKAP12-related immunomodulators were involved in important functions related to tumorigenesis and development (Figure 4(b)). Pathway enrichment volcano map showed that significantly enriched pathways of AKAP12-related immunomodulators include some immune and tumor-related pathways (Figure 4(c)).

The article "Comprehensive Analysis of the Immune Implication of AKAP12 in Stomach Adenocarcinoma" was published in 2022. Journal: Comput Math Methods Med.

### 3.4. Construction of an AKAP12-Related Immunomodulator Prognostic Signature

To investigate the prognostic significance of the AKAP12-related immunomodulators, the expression profile of 46 candidate AKAP12-related immunomodulators combined with survival data was analyzed in TCGA-STAD dataset (*n* = 371) using a stepwise multivariate Cox regression analysis. Through filtration with *p* value < 0.05 as the cutoff in univariate Cox regression analysis, 7 of 46 AKAP12-related immunomodulators were identified to be associated with the overall survival of patients (Figure 5(a)). Then, a prognostic risk signature containing four AKAP12-related immunomodulators (CXCR4, IL6, NT5E, and TNFSF18) was constructed following stepwise multivariate Cox regression analysis (Figure 5(b)). In this prognostic signature, each patient risk score was calculated through the proposed formula: risk score = sum of the expression level of the four immunomodulators × their respective coefficient. Patients were then divided into high- and low-risk groups according to the optimal risk score cutoff. Survival curve exhibited that the high-risk group patients had a worse prognosis than the low-risk group patients, with *p* value < 0.001 (Figure 5(c)). The risk heat map displayed the expression of the four risky immunomodulators was upregulated as the patient's risk score increased, and the high-risk group also had higher deaths than the low-risk group (Figure 5(d)). Then, we aimed to test whether the risk signature was independent of other clinicopathological characteristics; our results showed that the risk score was significantly associated with overall survival following the univariate Cox regression analysis (HR = 2.128, 95%CI = 1.549–2.922, and *p* value < 0.001) (Figure 5(e)). Moreover, with correction for age, gender, grade, and stage in the multivariate Cox regression model, we found that the risk score still retained its prognostic significance as an independent prognostic factor for STAD patients (HR = 1.863, 95%CI = 1.318–2.634, and *p* value < 0.001) (Figure 5(f)). Furthermore, the receiver operating characteristic (ROC) curve showed that risk signature had an area under the curve (AUC) value of 0.652 (Figure 5(g)). Finally, we generated a nomogram to evaluate the predicting performance of the risk score combined with other clinical factors in TCGA-STAD patients (Figure 6(a)). The concordance index (C-index) that reflects the accuracy of prediction and actual survival situation was 0.608. The calibration curve displayed that the predicted probability of the nomogram (red line) closely matched the ideal reference line (gray line) for the 5-year survival prediction (Figure 6(b)).

The article "Comprehensive Analysis of the Immune Implication of AKAP12 in Stomach Adenocarcinoma" was published in 2022. Journal: Comput Math Methods Med.

## 4. Discussion

STAD is one of the malignant tumors that endanger human health. For early STAD, surgery combined with chemotherapy has a significant effect, but for advanced STAD, its effect is not ideal [33]. Immunotherapy provides hope for the treatment of patients with advanced STAD, but there is a defect in drug resistance [12]. Thus, it is essential and urgently needed to identify novel biomarkers of immunotherapy in STAD. In the present study, we systematically analyzed the immune significance of the tumor suppressor AKAP12 from various aspects including immune infiltration cells, immune-related pathways, and immunomodulators and constructed an AKAP12-related immunomodulator prognostic signature. Our results suggest that AKAP12 may be a potential immunotherapeutic target for STAD.

The regulatory effect of AKAP12 as a tumor suppressor gene in tumors has been extensively studied and confirmed. For instance, KAP12 expression is downregulated in colorectal tumor tissues, and AKAP12 methylation level was positively associated with tumor grade [16]. Exogenous overexpression of AKAP12 in Lovo colon cancer cell line inhibits tumor cell proliferation, migration, and invasion ability [18]; in contrast, AKAP12 silencing or AKAP12/HDAC3 cosilencing promotes tumor cell proliferation, colony-forming ability, and cell cycle progression [20]. These studies suggest AKAP12 plays a protective role in preventing the occurrence and progression of colorectal cancer. In addition to its inhibitory effect on tumor growth and metastasis by scaffolding key regulatory proteins such as protein kinase C, F-actin, and cyclins, AKAP12 also exerts important role in the drug resistance mechanism of tumors [14, 15, 34]. In our present study, we also detected a significantly lower expression of AKAP12 in STAD. Moreover, CpG island hypermethylation was frequently observed in the promoter region of AKAP12 in gastric cancer, and the expression of AKAP12 can be restored through methyltransferase inhibitor [17], suggesting DNA methylation is directly involved in the silencing of the AKAP12 in gastric cancer. Furthermore, the reexpression of AKAP12 in gastric cancer cell line induced apoptotic cell death and reduced colony formation [17], indicating AKAP12 is a potential tumor suppressor of gastric cancer.

The article "Comprehensive Analysis of the Immune Implication of AKAP12 in Stomach Adenocarcinoma" was published in 2022. Journal: Comput Math Methods Med.

Tumor immunotherapy reflects the complex cellular and molecular interactions between tumor cells and the surrounding immune microenvironment [21]. An important content of our research is to clarify the association between AKAP12 and immune infiltration cells in STAD. Based on TIMIR database, our results demonstrated that AKAP12 expression was positively related to CD4^+^ T cells and macrophages. Besides that, the deletion of AKAP12 somatic copy number causes a reduction in the infiltrating proportion of B cell, CD8^+^ T cell, CD4^+^ T cell, and dendritic cell. It should be noted that the abovementioned immune cells are a fuzzy classification concept. It is essential to investigate the precise tumor-promoting or -suppressing immune cells to clarify the specific role of AKAP12-related immune cells. For this purpose, CIBERSORT algorithm containing 22 types of infiltrating immune cells was performed, and the results showed the infiltrating abundance of tumor-suppressing immune cells, such as native B cells, memory resting CD4 T cells, and activated NK cells, was significantly higher in patients with AKAP12-high expression. These results suggest that AKAP12 may play an important effect on immune cell infiltration of STAD.

Furthermore, our results confirmed that AKAP12 is involved in the regulation of immune-related signaling pathways from at least three perspectives. Firstly, KEGG pathway analysis in our study revealed that AKAP12 coexpressed genes were significantly enriched in PI3K-Akt signaling pathway and mTOR signaling pathway. It is well established that the PI3K-AKT-mTOR signaling network is dysregulated in human cancer, and PI3K-AKT-mTOR inhibitors can not only target cancer cell biology but also weaken immune cell effector functions [35, 36]. Secondly, GSEA enrichment analysis in our study showed that antigen processing and presentation are activated in patients with AKAP12 high expression, which has been proved to be an important and essential link in the process of immune cells killing cancer antigens in tumor immunity [37]. Thirdly, KEGG pathway analysis based on AKAP12-related immunomodulators demonstrated that several important immune pathways including Th17 cell differentiation and natural killer cell-mediated cytotoxicity were involved in AKAP12-mediated immune events. Sun et al. reported that tumor exosomes promote Th17 cell differentiation and inhibit tumor growth by delivering lncRNA CRNDE-h in colorectal cancer [38]. Shen et al. provide evidence that natural killer cell-mediated cytotoxicity can be enhanced to kill breast cancer cells by silencing NKG2D ligand-targeting miRNA [39]. Taken together, we speculate that AKAP12 may also play an important role in gastric cancer tumor immunity through these immune-related pathways.

The article "Comprehensive Analysis of the Immune Implication of AKAP12 in Stomach Adenocarcinoma" was published in 2022. Journal: Comput Math Methods Med.

In recent years, as ICI have made breakthroughs in the treatment of gastric cancer, and more and more immune-related gene signatures have been identified to evaluate the prognosis of gastric cancer patients. For example, Wang et al. identified a stromal-immune score-based 4-gene prognostic signature by estimating stromal and immune scores from TCGA and Gene Expression Omnibus (GEO) gastric cancer data [40]. Liu et al. developed an immune-related gene pair signature based on ImmPort database, and the signature is associated with overall survival and immune checkpoint expression in gastric cancer patients [41]. In our study, we also identified an AKAP12-related immunomodulator signature for STAD prognosis prediction, in which four immunomodulators (CXCR4, IL6, NT5E, and TNFSF18) were included. CXCR4 encodes a CXC chemokine receptor specific to stromal cell-derived factor-1, which has seven transmembrane regions and is located on the cell surface. The cases studied by Kamihara et al. [42] indicated that CXCL12 (SDF-1)/CXCR4 axis is involved in the observed metastasis of diffuse large B cell lymphoma to primary STAD and considered that the interaction between chemokines and their receptors may be the potential mechanism of the observed metastasis between tumors. IL6 encodes a cytokine that plays a role in inflammation and B cell maturation. The study of Ju et al. [43] showed that tumor-associated macrophages through IL-6 and TNF-ɑ signal induce the expression of PD-L1 in gastric cancer cells and help tumor cells escape cytotoxic T cell killing. NT5E encodes a plasma membrane protein that catalyzes the conversion of extracellular nucleotides to membrane permeable nucleosides and performs many homeostatic functions in healthy organs and tissues. Since the free adenosine produced by NT5E can inhibit the cellular immune response and promote the immune escape of tumor cells, it can be used as an inhibitory immune checkpoint molecule [44]. TNFSF18 is a member of the tumor necrosis factor (ligand) superfamily 18 and has the activity of binding to tumor necrosis factor receptors. The results of Chen et al. showed that five differently expressed genes, including TNFSF18, can be used as a single biomarker to predict the efficacy of anti-PD-1 in patients with metastatic non-small-cell lung cancer [45]. In addition, this risk signature is not only an independent prognostic factor for gastric cancer but also presents good prediction performance. Moreover, we provide a reference for the individualized prognosis of patients by integrating the risk score and other clinical factors to construct a nomogram.

The article "Comprehensive Analysis of the Immune Implication of AKAP12 in Stomach Adenocarcinoma" was published in 2022. Journal: Comput Math Methods Med.

In conclusion, despite the flaws in our study, for example, pure bioinformatics analysis without experimental verification, our study provides strong evidence that AKAP12 is closely related to tumor immunity in STAD from three aspects: immune infiltration cells, immune pathways, and immunomodulators. More importantly, the AKAP12-related prognostic signature may provide good application prospects for clinical practice.

## Figures and Tables

**Figure 1:** The expression of AKAP12 in STAD and its relationship with immune infiltrating cells. (a) The mRNA expression levels of AKAP12 in TCGA-STAD tissues and normal samples. ^∗∗^*p* < 0.01. (b) Immunohistochemical analysis of AKAP12 protein expression in STAD and normal tissues. Data were obtained from HPA database. The brown areas represent positive expression and the blue negative. (c) Correlation analysis between AKAP12 mRNA expression and six types of immune infiltrating cells based on TIMER database. The relation coefficient and *p* value are shown in each plot. (d) Associations between AKAP12 gene copy numbers and immune cell infiltration levels based on TIMER database. The *p* value is shown in each plot. (e) Violin plot displaying the infiltrating levels of 22 types of immune cells between the AKAP12^high^ expression group and the AKAP12^low^ expression group (group cutoff = AKAP12 expression median). The *p* value is shown in the figure.

**Figure 2:** AKAP12 is associated with cancer- and immune-related pathways based on CCLE project. (a) GO function annotation based on AKAP12 coexpressed genes. (b) KEGG pathway analysis based on AKAP12 coexpressed genes. (c) GSEA enrichment analysis of AKAP12^high^ and AKAP12^low^ expression groups.

**Figure 3:** Identification of AKAP12-associated immunomodulators in STAD. (a) Correlation heat map and dot plots showed 15 immunoinhibitors significantly associated with AKAP12 expression in STAD. (b) Correlation heat map and dot plots showed 31 immunostimulators significantly associated with AKAP12 expression in STAD.

The article "Comprehensive Analysis of the Immune Implication of AKAP12 in Stomach Adenocarcinoma" was published in 2022. Journal: Comput Math Methods Med.

**Figure 4:** Analysis of the pathways involved in AKAP12-associated immunomodulators. (a) Constructing a PPI network based on the 46 AKAP12-associated immunomodulators using STRING tool. (b) GO function annotation based on the 46 AKAP12-associated immunomodulators using WebGestalt online tool. (c) KEGG enrichment analysis based on the 46 AKAP12-associated immunomodulators using WebGestalt online tool.

**Figure 5:** Construction of a prognostic gene signature based on AKAP12-associated immunomodulators. (a) The associations between AKAP12-associated immunomodulators and overall survival in STAD using univariate Cox regression analysis. (b) The hazard ratios of AKAP12-associated immunomodulators integrated into the prognostic signatures are shown in the forest plots for TCGA-STAD patients. (c) Survival curve for risk score based on Kaplan–Meier analysis in TCGA-STAD patients. (d) Distribution of risk scores, survival status, and gene expression profiles for the TCGA-STAD patients. (e) Univariate and (f) multivariate Cox regression analyses of the risk score and overall survival in TCGA-STAD patients. (g) Time-dependent ROC curve for the risk score in TCGA-STAD patients.

**Figure 6:** Prognostic nomogram for TCGA-STAD dataset. (a) Nomogram for predicting the overall survival of TCGA-STAD patients. (b) Calibration curves of 1-, 3-, and 5-year overall survival of TCGA-STAD patients. Red line: nomogram-predicted survival curve. Gray line: ideal survival reference curve.

## Data Availability

The datasets generated and/or analyzed during the current study are available from the corresponding author on reasonable request. Data used included The Cancer Genome Atlas (TCGA, http://portal.gdc.cancer.gov/projects).

## Abbreviations

AKAP12: A kinase anchor protein 12
AUC: Area under the curve
CCLE: Cancer Cell Line Encyclopedia
CIBERSORT: Cell-Type Identification by Estimating Relative Subsets of RNA Transcripts
C-index: Consistency index
CNA: Copy number alterations
dMMR: Different mismatch repair
FDR: False discovery rate
GEO: Gene Expression Omnibus
GO: Gene Ontology
GSEA: Gene Set Enrichment Analysis
HPA: Human Protein Atlas
ICI: Immune checkpoint inhibitors
KEGG: Kyoto Encyclopedia of Genes and Genomes
MSI-H: Highly microsatellite instability
PD-1: Programmed cell death 1
PD-L1: Programmed cell death ligand 1
PPI: Protein-protein interaction
ROC: Receiver operating characteristic
STAD: Stomach adenocarcinoma
TCGA: The Cancer Genome Atlas
TIMER: Tumor Immune Estimation Resource
WebGestalt: Web-Based Gene Set Analysis Toolkit.
